The article "The preferences of 600 patients for different descriptions of randomisation" was published in 2005. Journal: Br J Cancer.

# The preferences of 600 patients for different descriptions of randomisation

**DOI:** 10.1038/sj.bjc.6602445

**Published:** 2005-02-22

**Authors:** V Jenkins, L Fallowfield, A Cox

**Affiliations:** 1 Cancer Research UK Psychosocial Oncology Group, Brighton and Sussex Medical School, University of Sussex, Falmer, East Sussex, BN1 9QG, UK

**Keywords:** randomisation, patients' preferences

## Abstract

A total of 600 patients from cancer centres throughout the UK identified their most preferred and most disliked descriptions of randomisation found in current patient information sheets and websites. The CancerBACUP description, which describes both the process of randomisation and why it is done, was most preferred 151 out of 533 (28%) patients. The NCI description was viewed as overly technical and most disliked 185 out of 483 (38%) patients.

There is an increasing expectation that patients should participate actively in decision making and evidence that properly informed patients are more likely to adhere to treatment (Epstein *et al*, 2004); thus, communicating clearly with patients and their relatives is paramount. One discussion that challenges many health professionals, even those with previous training in general communication skills (Jenkins *et al*, in press), is talking about randomised clinical trials (RCTs). The trial dialogue has many aspects that must be explained clearly and be tailored to an individual's needs and level of understanding to enable educated decision making. Random allocation of treatment is a key feature that patients have to appreciate prior to giving informed consent (Robinson *et al*, 2004).

The concept of randomisation produces difficulties for both patients and health professionals (Featherstone and Donovan, 1998, 2002; Fleissig *et al*, 2001; Kerr *et al*, 2004; Robinson *et al*, 2004; Simon *et al*, 2004) and among members of the public (Corbett *et al*, 1996; Kerr *et al*, 2004; Robinson *et al*, 2004). A series of studies exploring lay conceptions of the scientific and ethical justifications for random allocation and equipoise showed that while most participants could correctly identify whether or not a method such as tossing a coin was random, they did not find randomisation itself acceptable nor that a clinician would not know which treatment was best (Kerr *et al*, 2004; Robinson *et al*, 2004).

Although providing accurate ethical and understandable descriptions of randomisation is important, there is surprisingly little direct research elucidating the preferences of patients (Corbett *et al*, 1996; Featherstone and Donovan, 2002; Jenkins *et al*, 2002; Simon *et al*, 2004).

Patient information sheets about RCTs describe the randomisation process in a variety of ways, from ‘*allocate patients to a treatment group at random (this means by chance, a bit like drawing lots)*’ (TACT trial) (TACT – Standard anthracycline-based chemotherapy with fluorouracil, epirubicin and cyclophosphamide or epirubicin and CMF *vs* FEC followed by sequential docetaxel as adjuvant treatment for women with early breast cancer) ‘*randomisation means that neither you nor your doctor picks the treatment, but a computer will decide*’ (VICTOR trial) (VICTOR – double blind, placebo-controlled trial of rofecoxib in colorectal cancer patients following potentially curative therapy) to ‘*randomisation means that for each patient a computer will be used in the central office in London at the Medical Research Council Trials Office to allocate by chance rather than a medical decision*’ (REO4 trial) (RE04 – a trial of interferon-*α*, interleukin-2 and 5-fluorouracil *vs* interferon-*α* alone in advanced renal cell cancer). Explanations such as ‘*drawing lots’* might sound somewhat chancier than phrases such as *‘a computer will decide*’, but suggesting that a computer will decide may subtly mislead patients into believing that a considered decision based on their individual clinical details will be made.

The article "The preferences of 600 patients for different descriptions of randomisation" was published in 2005. Journal: Br J Cancer.

In a previous survey, the preferences of 200 cancer patients and 341 members of a healthy lay population were compared with the most commonly used descriptions of 200 oncologists. The study used the seven simulated descriptions of randomisation taken from the only other publication on the subject at the time (Corbett *et al*, 1996). Results showed that one explanation did not suit all. Analogies for allocation of treatment such as a *‘toss of a coin’* were disliked by 31% of patients and almost a quarter of the public, although this was a favoured description used by 26% clinicians in the survey (Jenkins *et al*, 2002). The primary limitations of this publication was that it utilised the contrived descriptions employed by the original Corbett study (Corbett *et al*, 1996). In an effort to further inform health professionals, we performed another preference survey using seven actual descriptions of randomisation.

## MATERIALS AND METHODS

### Descriptions

The authors reviewed over 100 definitions of randomisation taken from current patient information sheets and information websites. From these, seven were chosen which provided a broad range of those in frequent use (see Table 1). Presentation order of the descriptions was varied in a balanced manner to prevent any bias due to the effects of order. Patients were not aware of the origin of each description.

### Questionnaire

Patients read the following short scenario:

*‘Imagine that you have an appointment with a specialist to talk about how to treat your condition. The specialist tells you there is a research trial going on in the hospital comparing different treatments that are suitable for your illness. However, the only scientific way to compare one treatment with another is for the choice between the treatments to be made randomly’.*

The article "The preferences of 600 patients for different descriptions of randomisation" was published in 2005. Journal: Br J Cancer.

Patients were then asked to rate whether they found each description ‘unclear’, ‘fairly clear’ or ‘very clear’, to indicate their most preferred and disliked statement and then provide a reason for their choice if they wished.

### Sample

The questionnaire probed basic demographic details such as age, sex, cancer site and previous trial experience but was anonymous. In total, 43 doctors and nurses from 24 oncology centres across the UK who had attended a communication in clinical trials course were invited to distribute questionnaires to unselected patients with cancer aged over 18 years attending their outpatient clinics. Each questionnaire was attached to an information sheet with a stamped addressed envelope. A total of 1128 questionnaires were provided to healthcare professionals; of these, 600 were returned giving a 53% response rate. This figure might be an underestimate, as it is not known if all the questionnaires were actually administered. The patient demographics are shown in Table 2.

The study had full MREC and R&D approvals.

### Statistics

Statistical Package for the Social Sciences (SPSS) version 11.5 was used for all statistical analyses.

## RESULTS

### Clarity of descriptions

Most patients indicated that descriptions were fairly or very clear, percentages are shown in Table 3. There were no significant differences in clarity ratings by age, sex, previous trial experience or sociodemographic characteristics.

### Preferred description

The *χ*^2^ analysis showed a significant difference both for preference and dislike across the descriptions (preferred *X*^2^=199.74, df=6, *P*<0.0001; disliked *X*^2^=251.22, df=6, *P*<0.0001). Table 3 displays the frequency counts of preferences for each statement, 497 patients nominated both their most preferred and most disliked descriptions, two patients disliked all of them, 56 did not express any preference, 36 only nominated a preferred description and 10 patients gave only their most disliked description.

The most preferred description was that found on the CancerBACUP website (28% (151 out of 533)). Reasons patients gave for their choice included *‘it explains how and why’*, *‘it explains why treatment is randomly allocated to patients’* and *‘it sounds as if there is a sense and a meaning for the computer choosing a treatment’.* Also, this description was one of only two that did not mention the word ‘chance’ or use an analogy for chance. It also explains the need for randomisation that is the prevention of bias. Significant numbers of patients also favoured the descriptions on the Royal Marsden website (20% (106 out of 533)) and that given in the MRC Focus Trial information sheet (19% (101 out of 533)).

The article "The preferences of 600 patients for different descriptions of randomisation" was published in 2005. Journal: Br J Cancer.

### Most disliked description

Description 3 from the National Cancer Institute (NCI) website was the most disliked (38% (193 out of 508)) and this was consistent regardless of cancer site, age, previous trial experience or sociodemographic characteristics. This is one of the shortest descriptions but was repeatedly criticised by patients for using unfamiliar language and terminology *‘too technical’, ‘used long complicated words and terms’* and *‘its use of language assumes knowledge of the research process’.*

## DISCUSSION

Explaining clearly the concept of randomisation is fundamental to ensuring properly educated consent to clinical trial participation, yet studies have shown that despite different verbal and written explanations, patients still remain confused and unclear about the phrases used (Featherstone and Donovan, 2002; Simon *et al*, 2004).

In the survey reported here, most descriptions in current use are viewed as clear, but patients have preferences for some rather than others. The CancerBACUP website (2003) provided the most preferred description of randomisation irrespective of age, sex or cancer site and previous trial experience, while that found on the NCI website (2003) was the most disliked description.

In contrast to our previous study, the description that included the analogy ‘toss of a coin’ did not produce such fervent dislike by the majority of patients (Jenkins *et al*, 2002). One explanation is that the analogy did not stand alone, it was prefaced by the statement that a computer would choose *‘like the toss of a coin’* together with an explanation that it is done to prevent bias. Patients who did dislike it expressed similar comments to those found in the previous survey such as *‘My life should not depend on the ‘toss of a coin’, ‘the roll of a dice’ or chance.’*

The NCI description found favour with a mere 17 (3%) of the sample and overshadowed all others for dislike. In particular, patients did not like the use of what they felt was jargon and several commented that, *‘the English was a bit too complex’*.

Given the multinational nature of many RCTs and a desire for uniformity of patient information accompanying them, some crosscultural research on descriptions of randomisation might be warranted. The language in the description from an American website was especially disliked by UK patients, which could produce a potential barrier to participation in trials.

The article "The preferences of 600 patients for different descriptions of randomisation" was published in 2005. Journal: Br J Cancer.

## Figures and Tables

**Table 1:** Descriptions of randomisation

1	Once you have agreed to enter the trial, your treatment is not chosen by yourself or a doctor but by a computer. There is usually a 50 : 50 chance of receiving either treatment	Royal Marsden Website, 2003
2	Once you have agreed to enter the trial, a computer will allocate you randomly (as if by the roll of a dice) to receive the ‘standard treatment’ or one of the new treatments being tested. Neither your doctor nor you yourself will choose which treatment you receive	MRC FOCUS Trial Patient info sheet
3	Once you have agreed to enter the trial, you will be randomised to a course of treatment. This is a process that assigns participants by chance, rather than by choice, to either the investigational group or the control group	NCI website, 2003
4	Once you have agreed to enter the trial the decision regarding which treatment you receive will be made by a process called ‘randomisation’. This means that your specialists will not make the decision themselves, but it will be made by chance	BNL Trial Patient info sheet
5	Once you have agreed to enter the trial, the treatment you receive will be selected by a process called randomisation, that is, it will not be chosen by you or your doctor, but by a computer and it is like the toss of a coin. This is to prevent bias in the results of the trial	CLL4 Trial Patient info sheet
6	Once you have agreed to enter the trial, you will be randomised to a course of treatment. This means that there are at least two different groups in the trial and those taking part are put into one or other group at random. This ‘randomisation’ is usually done by a computer	CancerHelp website, 2003
7	Once you have agreed to enter the trial, you will be randomised to a course of treatment. This means that a computer will randomly allocate patients to treatment groups in the trial. This is done so that each group has a similar mix of patients of different ages, sex and state of health	CancerBACUP website, 2003

**Table 2:** Patient demographic information

	***N*=600**	**(%)**
*Sex*		
Male	226	37.7
Female	337	56.2
Missing	37	6.2
		
*Previous trial experience*	169	28.2
		
*Age*		
Under 60 years	298	49.7
60 years and over	273	45.5
Missing	29	4.8
		
*Cancer site*		
Breast	220	36.7 (*15*)
GI/colorectal	76	12.7 (*16*)
Gynaecological	33	5.5 (*6*)
Lung	30	5.0 (*14*)
Urological	121	20.2 (*15*)
Haematological	35	5.8 (*6*)
Muscular/skeletal	22	3.7 (−)
Brain	10	1.7 (*2*)
Other	21	3.5
Missing	32	5.3
		
*Regions of UK*		
Southern England (inc. London)	295	49.25
Midlands	74	12.35
Northern England	110	18.4
Scotland	47	7.8
Wales	73	12.2
Missing	1	

*N* italics, UK incidence (CRUK, 2001).

The article "The preferences of 600 patients for different descriptions of randomisation" was published in 2005. Journal: Br J Cancer.

**Table 3:** Showing frequency (%) of clarity ratings and preference/dislike for each statement

	**Overall clarity**				
**Statement**	**Very clear**	**Not at all/quite clear**	**Missing**	**Preference (*n*=533)**	**Dislike (*n*=508)**
1 Royal Marsden Website	361 (61)	236 (39)	3	106 (20)	69 (14)
2 MRC Focus trial	327 (55)	270 (45)	3	101 (19)	65 (13)
3 NCI Website	326 (55)	269 (45)	5	17 (3)	**193 (38)**
4 BNL Trial	335 (56)	260 (44)	5	23 (4)	62 (12)
5 CLL4 Trial	331 (56)	264 (44)	5	96 (18)	29 (6)
6 Cancer help website	325 (54)	272 (46)	3	39 (7)	53 (10)
7 Cancer BACUP website	333 (58)	258 (44)	9	**151 (28)**	37 (7)

Bold represents most preferred/most disliked.
